RETRACTED

# Bevacizumab Combined with Intensity-Modulated Radiation Therapy on Cognitive and Coagulation Function in Postoperative Glioma Patients

**DOI:** 10.1155/2022/9367919

**Published:** 2022-03-12

**Authors:** Guo-Shi Lin, Wei-Wei Wang, Hong Lin, Rui-Sheng Lin

**Affiliations:** Department of Neurosurgery, Zhangzhou Affiliated Hospital of Fujian Medical University, Zhangzhou, Fujian 363000, China

## Abstract

To examine the influences of bevacizumab combined with intensity-modulated radiation therapy (IMRT) on postoperative brain glioma, particularly its impact on coagulation function and cognitive function, the complete clinical data of 156 patients undergoing glioma surgery in the neurosurgery department of our hospital between March 2015 and October 2018 were retrospectively analyzed. All patients underwent glioma surgery and were then assigned to the observation group (Obs group, *n* = 79, received bevacizumab combined with IMRT) or the control group (Con group, *n* = 77, received IMRT without bevacizumab) for analysis during postoperative treatment. The patients' short-term efficacy was evaluated, and their serum markers and coagulation function were compared, as well as the cognitive function, the occurrence of adverse reactions during treatment, the Karnofsky performance status (KPS) score, and quality of life after treatment. Patients' survival was followed up within 2 years after surgery. The Obs group showed a notably higher clinical remission rate and clinical control rate (DCR) than the Con group after treatment. The Obs group showed notably lower levels of interleukin-2 (IL-2), vascular endothelial growth factor (VEGF), IL-6, and epidermal growth factor (EGF), experienced notably shorter prothrombin time (PT) and activated partial thromboplastin time (APTT), and showed higher fibrinogen (FIB) and D-dimer (D-D) levels than Con group. The Obs group showed notably better cognitive function, KPS score, and quality of life than the Con group, but no notable difference was observed between them in the incidence of adverse reactions (*P* > 0.0500). The survival rates in the Obs group were higher than in the Con group. For patients with glioma, postoperative bevacizumab combined with IMRT delivers substantially higher clinical efficacy by lowering serum marker levels and improving cognitive function without significantly affecting coagulation function.

## 1. Introduction

Glioma is a frequently seen primary intracranial brain tumour, and its pathological types include astrocytoma, oligodendroglioma, ependymoma, and mixed glioma, of which astrocytoma is the most frequently seen one [1]. Glioma is characterized by high incidence, recurrence, and mortality [2]. Clinical symptoms mainly include increased intracranial pressure, neurological dysfunction, cognitive dysfunction, seizures, etc. [3]. Glioma is more frequently seen among individuals above 40 years old, with a higher incidence among the elderly over 60 years old. The World Health Organization classifies gliomas into grades I–IV at the pathological level, of which grades I-II and grades III-IV are considered as low-grade gliomas and high-grade gliomas, respectively [4]. Low-grade gliomas have relatively better prognosis than high-grade gliomas, with an overall survival period of about 5–10 years, but about 30% of low-grade gliomas recurrence can further malignant lesions to higher pathological grades glioma [5]. The treatment effect of high-grade glioma is very unsatisfactory, among which glioblastoma has a median survival time of only 18 months and 5-year survival time lower than 10% [6].

RETRACTED

At the current stage, surgical resection is still the preferred therapy for glioma [7], whereas, due to the characteristics of invasive growth of gliomas, the boundary of tumour lesions in cases with low-grade or high-grade gliomas is not clear, and it is difficult to completely remove the lesions by surgery, especially high-grade gliomas. The main mode after treatment failure is local recurrence [8]. In order to kill residual glioma, prevent postoperative recurrence, and reduce postoperative recurrence rate, patients with glioma often take adjuvant radiotherapy after surgery. Intensity modulated radiotherapy (IMRT) is a commonly used adjuvant method to kill residual cancer cells and prevent tumour recurrence in recent years [9]. IMRT has the characteristics of precise localization and can adjust the irradiation dose of the target region according to the shape and position of the tumour. While killing the cancer cells, it can minimize the radiation damage to the surrounding normal tissues and effectively control the growth, metastasis, and diffusion of the tumour [10, 11]. However, due to the poor sensitivity of glioma to radiotherapy, the postoperative IMRT alone has very limited preventive value for recurrence.

At the same time, recent research has indicated the high level of vascular endothelial growth factor (VEGF) as one crucial factor promoting tumour invasive growth [12]. Therefore, from this perspective, it is a new idea to use drugs that antagonize the biological function of VEGF for combination therapy. Bevacizumab has been approved by the US Food and Drug Administration as one antivascular agent for the therapy of recurrent high-grade gliomas [13]. However, there are some concerns with the use of bevacizumab, including the potential for tumour hemorrhage and venous thrombosis [14]. Now, studies on coagulation function and cognitive function of patients after glioma with bevacizumab combined with IMRT have not been reported. From the perspective of coagulation function and cognitive function, this study retrospectively analyzed the impacts of bevacizumab + IMRT on postoperative patients with glioma and its impacts on cognitive function and coagulation function, providing more evidence for clinical treatment of glioma.

RETRACTED

## 2. Materials and Methods

### 2.1. Subjects

The complete clinical data of 156 patients undergoing glioma surgery in the neurosurgery department of our hospital between March 2015 and October 2018 were retrospectively analyzed. All patients continued to receive treatment postoperatively, with the choice of treatment initially based on patient willingness to undergo surgery and individual patient circumstances. In the light of different treatment means, patients were assigned to the control group (Con group, receiving postoperative intensity modulated radiation therapy, *n* = 77) and observation group (Obs group, receiving postoperative bevacizumab combined with intensity modulated radiation therapy, *n* = 79). This study was carried out under the ethical standards of clinical trials and approval of the hospital's Medical Ethics Committee (Approval number: 2021KYB203).

### 2.2. Inclusion and Exclusion Criteria

The inclusion criteria were as follows: (1) all with typical clinical manifestations such as headache and vomiting, loss of vision, and a clear diagnosis of glioma and treated with surgical resection, pathological grade III-IV; (2) all who started radiotherapy after the healing of the surgical incision (2–4 weeks); (3) age <80 years and expected survival >3 months; (4) Karnofsky (KPS) score ≥60; (5) those who had not been previously treated with any of the drugs used in this study; (6) complete clinical information.

Exclusion criteria were as follows: (1) patients with contraindications of surgery, radiotherapy, or allergy to drugs used in this study; (2) patients who have received chemotherapy or head and neck tumour sensitization radiotherapy; (3) presence of other cranial diseases or other serious pathological changes of tissues, organs, and systems; (4) poor treatment coordination, mental disorders; (5) incomplete clinical information.

### 2.3. Treatment Protocol

In both groups, intensity modulated conformal radiotherapy was performed with 6MV-X radiation at 2–4 weeks after surgery: Each patient was required to lie in a comfortable supine position to make a U-shaped thermoplastic mask for the head, and the head frame and thermoplastic mask were used to fix the position. According to CT and MRI examination results of patients before and after surgery, the lesion status was determined and target areas were marked, which were divided into tumour target area (GTV), clinical target area (CTV), and planned target area (PTV). Residual lesions in T1-weighted enhanced images, abnormal signals in water-inhibited T2, and intraoperative cavity were assigned as GTV1, residual lesions in T1-weighted enhanced images and intraoperative cavity were assigned as GTV2, and residual lesions in T1-weighted enhanced images were assigned as GTVp. CTV1 was obtained by GTV1 extending 1.5–2.0 cm outward. PTV1 was obtained by CTV1 expanding 0.3–0.5 cm outwards, CTV2 by GTV2 expanding 1.0–1.5 cm outwards, and PTV2 by CTV2 expanding 0.3–0.5 cm outwards. Radiotherapy dose: PTV1 was 54 Gy/30 times, PTV2 was 60 Gy/30 times, and CTV was 642–66.0 Gy/30 times. The segmentation dose was 1.8 Gy for PTV1, 2.0 Gy for PTV2, and 2.14–2.20 Gy for CTV, five times a week.

RETRACTED

The Obs group was treated with bevacizumab in addition to IMRT, and bevacizumab was intravenously injected into 500 mL normal saline with 5–10 mg/kg bevacizumab every 2 weeks for 3 months (about 6 cycles).

### 2.4. Observation Indicators

1. Short-term efficacy assessment: Three months after the end of radiotherapy, all patients underwent imaging examinations. Based on the Response Assessment in Neuro-Oncology (RANO) standard [15], the efficacy was classified into complete response (CR), partial response (PR), stable disease (SD), and progressive disease (PD). Clinical remission rate = (CR + PR)/total number of cases ×100%; clinical control rate = (CR + PR + SD)/total number of cases ×100%.
2. All patients received relevant hematological examination before radiotherapy and during follow-up. Serum marker detection: Fasting weekly venous blood was collected from each patient in the morning prior to treatment and 3 months after the end of radiotherapy, and the serum was separated for detection after standing at room temperature for natural coagulation and 20-min centrifugation (3000 r/min). Interleukin-2 (IL-2), IL-6, VEGF, and epidermal growth factor (EGF) were quantified using ELISA, with corresponding kits provided by Shanghai Enzyme-Linked Biotechnology Co., LTD. (article numbers: ml058063, ml058097, ml064281, and ml058660) under guidelines of the kits.
3. Coagulation function test: Venous blood was acquired from the elbow of every patient prior to radiotherapy and at 3 months after the end of radiation therapy and mixed with anticoagulant containing 0.109 mol/L sodium citrate (9 : 1), followed by 10-min centrifugation (3000 r/min) with shaking, and plasma was taken for measurement. The coagulation indexes, including prothrombin time (PT), prothrombin time (TT), fibrinogen (FIB), activated partial thromboplastin time (APTT), and fibrinolytic index (D-dimer, D-D), were measured through one automatic coagulation analyzer (STA-R Evolution, France).
4. Cognitive function assessment: All patients were assessed for cognitive function before surgery, before postoperative radiation therapy, and at the end of 3 months of radiation therapy using the Mini-Mental State Examination (MMSE) [16]. With a total score of 30 points, the main components included memory (3 points), orientation (10 points), recall (3 points), attention and calculation (5 points), and verbal ability (9 points). A higher score implies better cognitive function, and a total score of <27 suggests cognitive impairment.
5. Occurrence of adverse reactions and complications: During the treatment, intracranial pressure increase, gastrointestinal reaction, skin ulceration, bone marrow suppression, liver function injury, and other conditions were recorded in the 2 groups.
6. Health status and quality of life (QOL) score: The two groups were compared in the Karnofsky performance status (KPS) score [17] and QOL score [18] before and 3 months after radiotherapy. With a higher score implying better health, KPS scores are within 0–100, using 0 points for death and 100 points normal condition, without any symptoms or signs. QOL score includes 12 dimensions including appetite, pain, spirit, sleep, fatigue, understanding and cooperation of colleagues, own knowledge of cancer, attitude towards therapy, understanding and cooperation of family, daily life, facial expression, and adverse reaction to therapy. With a full score of 60, each dimension is divided into five grades. A lower score implies worse QOL: 51–60: very good, 41–50: good, 31–40: fair, 21–30: poor, and < 20: very poor.
7. Long-term survival rate: The 1-year and 2-year survival of patients were followed up from the date of surgery to December 2020, and the median survival inches were calculated.

RETRACTED

### 2.5. Statistical Methods

The normal approximation method in PASS 15.0 (NCSS Statistical Software, Kaysville, Utah) was adopted for the calculation of sample size. A preliminary analysis was conducted to the data at the level of bilateral test *α* = 0.0500. Assuming that the two-year survival rates of the Obs and Con groups were 74% and 50%, respectively, and 80% power was required, the sample size of each group was at least 61 cases, with 122 cases in total. Based on 20% loss rate, at least 77 cases should be included in each group, a total of 154 cases.

Statistical data were analyzed using SPSS 22.0 software package (IBM Corp., Armonk, NY, USA); GraphPad Prism 6.0 (GraphPad Software, La Jolla California USA) was used to visualize the data. Comparisons of count data [N (%)] were conducted via the *χ*2 test and fisher's exact test, and intergroup and introgroup comparisons of measurement data in normal distribution (Mean ± SD) were performed by independent sample *T* test and paired *T* test, respectively. We analyzed differences between groups at all time points (before surgery, before radiotherapy, and after radiotherapy) using repeated measures analysis of variance (ANOVA) and then the Bonferroni post hoc test. Kaplan–Meier analysis was applied to overall survival. With *α* = 0.0500 as test standard, *P* < 0.0500 implies a notable difference.

## 3. Results

### 3.1. Summary of Patients' General Baseline Information

No significant differences were identified in the patients' general baseline information between the control group and observation group (*P* > 0.0500), indicating a comparability (Table 1).

### 3.2. Short-Term Efficacy in Two Groups

The Obs group showed notably higher RR and DCR than the Con group 3 months after radiotherapy (all *P* < 0.0500, Table 2).

### 3.3. Changes of Serum Marker Levels in Two Groups

No notable difference was observed in the contents of IL-2, IL-6, VEGF, and EGF between the 2 groups before postoperative radiotherapy (*P* > 0.0500), while 3 months after radiotherapy, the contents of them in both groups dropped notably, with greatly lower levels in the Obs group than those in the Con group (all *P* < 0.0500, Figure 1).

### 3.4. Changes in the Coagulation Indexes of Two Groups

The two groups were similar in TT before and after radiotherapy (*P* > 0.0500). Three months after radiotherapy, both groups experienced notably shortened PT and APTT and showed notably increased FIB and D-D contents, with notably shorter PT and APTT and notably higher FIB and D-D contents in the Obs group than those in the Con group (all *P* < 0.0500, Table 3).

### 3.5. Cognitive Functions

Attention, memory, orientation, and computation, language ability, recall ability, and MMSE total score of the two groups before postoperative radiotherapy were notably higher than those before surgery (*P* < 0.0500), without notable difference between the 2 groups (*P* > 0.0500). Three months after the end of radiotherapy, the scores of all indicators of cognitive function and the total MMSE scores of the two groups elevated notably, with notably higher scores of all indicators and the total MMSE scores in the Obs group than those in the Con group (*P* < 0.0500, Table 4).

### 3.6. Occurrence of Adverse Reactions

The Obs group had 35, 2, 9, and 3 cases of gastrointestinal reaction, skin ulceration, bone marrow suppression, and liver function injury, respectively, with a total incidence of 62%. The Con group had 32, 3, 8, and 2 cases of gastrointestinal reactions, skin ulceration, bone marrow suppression, and liver function injury, respectively, with a total incidence of 58.4%. The two groups were similar in the incidence and total incidence of adverse reactions (*P* > 0.0500, Table 5).

RETRACTED

### 3.7. KPS Score and QOL

No notable difference was observed between the two groups in KPS and QOL scores before radiotherapy (*P* > 0.0500). KPS and QOL scores in both groups greatly increased 3 months after radiotherapy (*P* < 0.0500), with notably higher KPS score and QOL score in the Obs group than those in the Con group (*P* < 0.0500, Figure 2).

### 3.8. Long-Term Survival

The Obs group showed notably higher 2-year survival rates than the Con group (*P* < 0.0500, Figure 3).

## 4. Discussion

Infiltrating growth is the most prominent biological behavior of glioma, including infiltrating along white matter myelin fibers, nerve cells, and vascular tissue [19]. Since glioma cells migrate and grow invasive in the tumour area, surgical resection has limited efficacy for removing migrating tumour cells, and patients often relapse in a short period of time. However, surgical resection of partial lesions also enhances the efficacy of subsequent adjuvant therapy, prolonging the overall survival of patients to a certain extent. Postoperative radiotherapy is a conventional method to remove residual glioma lesions and prevent recurrence. Nevertheless, the long-term survival of postoperative radiotherapy alone is unsatisfactory. It is well known that solid tumour growth depends on continuous and extensive angiogenesis [20]. Glioma is a tumour rich in blood vessels. The new blood vessels caused by endothelial cell proliferation are closely related to the degree of biological invasion and malignancy of glioma [21]. Over the past few years, a large number of studies have pointed out the angiogenesis mediated by VEGF as a crucial link in the development of glioma [22]. Bevacizumab [23] is a targeted drug that specifically antagonizes VEGF and can produce biological effects that bind to VEGF and antagonize its promotion of angiogenesis. More and more data indicate that the combination of antiangiogenesis and chemoradiotherapy may improve the therapeutic effect [24]. This study was for clarifying the application value of bevacizumab + IMRT in cases with postoperative glioma. However, most previous studies focused on the overall survival of cancer treatment. With the progress of society, a growing number of people began to focus on the impact of cancer therapy on the QOL and physical function.

RETRACTED

In this study, we found notably higher overall efficacy, higher 1-year and 2-year survival rates, and longer median survival time in the Obs group than those in the Con group. These results suggested the ability of bevacizumab combined with IMRT in lifting the postoperative efficacy of glioma and prolonging the survival time of patients. We believed that bevacizumab may normalize tumour blood vessels and effectively reduce the hypoxic state in tumour while killing local tumour with IMRT, thus improving the efficacy of radiotherapy. Bevacizumab also selectively inhibits tumour-related angiogenesis and regeneration. After further analysis of the effect of bevacizumab, serum marker levels of patients were observed, and it was found that serum IL-2, IL-6, VEGF, and EGF in the 2 groups notably decreased after therapy, with notably lower levels in the Obs group than those in the Con group. Both IL-2 and IL-6 are cytokines that can promote the proliferation of tumour cells and the growth of vascular endothelial cells [25]. VEGF can directly act on endothelial cells and promote their proliferation to induce the formation of new blood vessels, while EGF can directly act on tumour cells to promote the growth of lesions [26]. These data implied that IL-6, IL-2, EGF, and VEGF produced in large quantities in the local lesions can be released into the blood circulation, and radiotherapy kills glioma cells and reduces the content of molecules related to proliferation activity in serum, but their effects were further enhanced with the addition of bevacizumab. All the above results indicate that bevacizumab combined with IMRT has stronger killing effect on tumour cells.

However, studies have found that the risk of deep vein thrombosis after brain tumour surgery is increased, which is mainly related to the secretion of hypercoagulable substances in the brain tissue during surgery [27]. Therefore, we detected the coagulation system function indicators of patients and found notably shorter PT and APTT and notably higher FIB and D-D contents in the Obs group than those in the Con group. Studies have pointed out that the shortening of APTT and PT indicates the hypercoagulable state of blood, which can be adopted for evaluating the risk of thrombosis and cardiovascular events in humans [28]. As a coagulation function protein molecule, FIB has the highest content in blood and is converted into fibrin catalyzed by thrombin, which affects the coagulation state in blood vessels. D-D, a specific degradation product of crosslinked fibrin, is also a specific indicator for secondary fibrinolysis evaluation and a major marker of thrombosis and hypercoagulability [29]. The increase of FIB and D-D indicates that the blood viscosity is elevated and thrombosis is likely to occur. Due to the injury of brain tissue in the process of surgery, a large number of tissue factors are secreted for activating the exogenous coagulation pathway of the body and eventually activating the endogenous coagulation pathway of the body, which is the disorder of the coagulation and anticoagulation system. However, with the addition of bevacizumab to the treatment, the incidence of abnormal coagulation function in patients increases, which has a certain risk. In addition, we found better improvement of cognitive function and higher KPS and QOL in the Obs group than those in the Con group. The results indicated that bevacizumab effectively improved the cognitive function and body function of patients. Patients with glioma are prone to postoperative complications of cerebral edema, which can affect cognitive function. Foreign literature has reported that bevacizumab can relieve radioactive brain edema and improve neurological function [30]. The results of this study also confirmed this point.

RETRACTED

## 5. Conclusion

The application of bevacizumab combined with IMRT effectively improves the short-term efficacy and survival rate of patients after glioma surgery, with significant clinical treatment effect and good application value and development prospect. However, this study also has limitations; the use time of bevacizumab in our study is not long-term. According to the results of this study, medium- and short-term use of bevacizumab can improve the curative effect of patients, but does long-term use have the same effect or is there any impact on the incidence of venous thrombosis? Therefore, the results of this study need further verification in randomized prospective studies with a larger sample size. In addition to coagulation function, the influencing factors on thrombosis should be comprehensively considered in combination with other factors such as patient age, tumour itself, chronic disease, and operation, so as to ensure the safe application of bevacizumab.

## Figures and Tables

**Figure 1:** Serum marker levels of two groups in different time points. (a) Comparison of IL-2 level between two groups before and after radiotherapy. (b) Comparison of IL-6 level between two groups before and after radiotherapy. (c) Comparison of VEGF level between two groups before and after radiotherapy. (d) Comparison of EGF level between two groups before and after radiotherapy. ^*∗∗∗*^*P* < 0.001 using paired *t*-test within group and independent sample *T* test between groups.

**Figure 2:** Intergroup comparison of KPS and QOL scores. (a) Comparison of KPS score between two groups before and after radiotherapy. (b) Comparison of QOL score between two groups before and after radiotherapy; ^*∗∗∗*^*P* < 0.001 using paired *t*-test within group and independent sample *T* test between groups.

RETRACTED

**Figure 3:** Kaplan–Meier analysis of 2-year overall survival.

**Table 1:** General baseline information (‾*x* ± *s*/*n*(%)).

	Control group (*n* = 77)	Observation group (*n* = 79)	*χ* ^2^/*t*	*P*
Gender [n(%)]			0.0219	0.8821
Male	41(53.2)	43(54.4)		
Female	36(46.8)	36(45.6)		
Average age (years,‾*x* ± *s*)	57.32 ± 6.43	58.02 ± 6.95	0.6526	0.5150
Pathological pattern			0.3095	0.8566
Neuroastrocytoma	47(61.0)	45(57.0)		
Oligodendroglioma	16(20.8)	19(24.1)		
Mixed glioma	14(18.2)	15(18.9)		
Lesion			1.2584	0.8685
Frontal lobe	32(41.6)	30(38.0)		
Occipital lobe	11(14.3)	14(17.7)		
Temporal lobe	19(24.7)	20(25.3)		
Parietal lobe	13(16.9)	11(13.9)		
Others	2(2.5)	4(5.1)		
Postoperative pathological grading			0.0855	0.7700
III	46(59.7)	49(62.0)		
IV	31(40.3)	30(38.0)		
Tumour diameter (cm,‾*x* ± *s*)	4.12 ± 0.87	4.02 ± 1.04	0.6506	0.5163
Degree of surgical resection			0.2059	0.6500
Complete excision	52(67.5)	56(70.9)		
Partial excision	25(32.5)	23(29.1)		
Combined underlying disease			0.2627	0.6083
Diabetes	15(19.5)	14(17.7)		
Hypertension	21(27.3)	25(31.6)		

Chi-square test, fisher's exact test, or independent sample *t*-test between groups.

**Table 2:** Intergroup comparison of short-term efficacy [n(%)].

Group	CR	PR	SD	*P*D	RR	DCR
Control group (*n* = 77)	9(11.7)	33(42.8)	22(28.6)	13(16.9)	42(54.5)	64(83.1)
Observation group (*n* = 79)	19(24.1)	42(53.1)	13(16.5)	5(6.3)	61(77.2)	74(93.7)
*χ* ^2^	10.5030				8.9341	4.2551
P	**0.0148**				**0.0028**	**0.0391**

Notes: CR: complete response; PR: partial response; SD: stable disease; PD: progressive disease; RR: response rate; DCR: disease control rate; chi-square test or fisher's exact test between groups. The bolded part represents statistical significance, *p* < 0.05.

**Table 3:** Comparison of coagulation indexes (‾*x* ± *s*).

Time point	Group	TT (s)	PT (s)	APTT (s)	FIB (g/L)	D-d (mg/L)
Before radiotherapy	Control group (*n* = 77)	17.85 ± 1.34	11.07 ± 1.17	24.52 ± 2.41	2.93 ± 0.31	0.32 ± 0.14
	Observation group (*n* = 79)	17.69 ± 1.43	11.32 ± 1.25	24.02 ± 2.49	3.01 ± 0.37	0.35 ± 0.11
t		0.7207	1.2889	1.2739	1.4619	1.4903
P		0.4722	0.1994	0.2046	0.1458	0.1382
3 months after radiotherapy	Control group (*n* = 77)	17.63 ± 1.56	10.18 ± 1.21^*∗*^	23.37 ± 2.51^*∗*^	3.41 ± 0.27^*∗*^	0.50 ± 0.13^*∗*^
	Observation group (*n* = 79)	17.52 ± 1.50	9.98 ± 1.04^*∗*^	21.05 ± 2.04^*∗*^	3.69 ± 0.35^*∗*^	0.59 ± 0.18^*∗*^
t		0.4489	1.9842	6.3427	5.5846	3.5723
P		0.6541	**0.0490**	<**0.0001**	<**0.0001**	**0.0005**

Notes: TT: thrombin time; PT: prothrombin time; APTT: activated partial thromboplastin time; FIB: fibrinogen; D-D : D-Dimer; *∗P* < 0.0500, compared to the same group before radiotherapy using paired *t*-test and independent sample *T* test between groups. The bolded part represents statistical significance, *p* < 0.05.

RETRACTED

**Table 4:** Comparison of cognitive functions (‾*x* ± *s*).

Time point	Group	Orientation	Registration	Calculation and attention	Recall	Language and visuospatial function	MMSE score
Before surgery	Control group (*n* = 77)	5.45 ± 0.51	1.50 ± 0.42	2.11 ± 0.39	1.11 ± 0.26	5.82 ± 0.85	21.23 ± 4.03
	Observation group (*n* = 79)	5.37 ± 0.42	1.53 ± 0.37	2.09 ± 0.32	1.17 ± 0.21	5.91 ± 0.77	21.59 ± 3.88
T		1.0707	0.4737	0.3505	1.5876	0.6934	0.5684
P		0.2860	0.6364	0.7264	0.1144	0.4891	0.5706
Before radiotherapy	Control group (*n* = 77)	7.74 ± 0.92^∗^	2.07 ± 0.40^∗^	3.12 ± 0.32^∗^	1.49 ± 0.27^∗^	7.03 ± 0.76^∗^	26.33 ± 2.05^∗^
	Observation group (*n* = 79)	7.86 ± 0.83^∗^	2.11 ± 0.36^∗^	3.17 ± 0.30^∗^	1.53 ± 0.22^∗^	7.10 ± 0.64^∗^	26.66 ± 2.07^∗^
T		0.8558	0.1099	1.0071	1.0156	0.6229	1.0002
P		0.3934	0.9127	0.3155	0.3114	0.5343	0.3188
3 months after radiotherapy	Control group (*n* = 77)	8.12 ± 0.77^∗#^	2.37 ± 0.40^∗#^	3.49 ± 0.29^∗^#	1.79 ± 0.31^∗#^	7.60 ± 0.74^∗#^	26.99 ± 1.89^∗#^
	Observation group (*n* = 79)	8.35 ± 0.64^∗#^	2.49 ± 0.32^∗#^	3.63 ± 0.33^∗#^	1.91 ± 0.23^∗#^	7.83 ± 0.68^∗#^	27.54 ± 1.16^∗#^
t		2.0310	2.0717	2.8119	2.7506	2.0222	2.1967
P		0.0440	0.0400	0.0056	0.0067	0.0449	0.0296

*Note.* ^∗^ *P* < 0.0500 *vs.* the same group before surgery; ^#^*P* < 0.0500 *vs.* the same group before radiotherapy; paired *t*-test and independent sample *T* test between groups.

**Table 5:** Adverse reactions in the two groups [n(%)].

Group	Gastrointestinal reaction	Skin eruptions	Myelosuppression	Hepatic injury	Total incidence rate
Control group (*n* = 77)	32(41.6)	3(3.8)	8(10.4)	2(2.6)	45(58.4)
Observation group (*n* = 79)	35(44.3)	2(2.5)	9(11.4)	3(3.8)	49(62.0)
*χ* ^2^	0.1199	0.2340	0.0404	0.1810	0.2091
P	0.7291	0.6286	0.8407	0.6705	0.6475

Chi-square test between groups.

## Data Availability

The clinical data used to support the findings of this study are included within the article.
